The article "Historical facts of screening and diagnosing diabetes in pregnancy" was retracted in 2014. Reasons: plagiarized text; overlap with other authors' work.

# Historical facts of screening and diagnosing diabetes in pregnancy

**DOI:** 10.1186/1758-5996-5-22

**Published:** 2013-05-01

**Authors:** Carlos Antonio Negrato, Marilia Brito Gomes

**Affiliations:** 1 Bauru’s Diabetics Association, Department of Internal Medicine, Bauru, São Paulo, 17012-433, Brazil; 2 Department of Internal Medicine, Diabetes Unit, State University Hospital of Rio de Janeiro, Rio de Janeiro, Brazil

**Keywords:** History of diabetes, Diabetes in pregnancy, Screening diabetes in pregnancy, Diagnosing diabetes in pregnancy

## Abstract

Diabetes is the most common metabolic disorder affecting pregnancy. Its prevalence seems to be growing in parallel with the epidemics of overweight and obesity. Recognizing and treating diabetes or any degree of glucose intolerance in pregnancy results in lowering maternal and fetal complications. These patients present higher risk for excessive weight gain, preeclampsia, cesarean sections, a high risk of developing type 2 diabetes and cardiovascular disease in the future. Infants born to these mothers are at higher risk for macrosomia and birth trauma, and after delivery, these infants have a higher risk of developing hypoglycemia, hypocalcemia, hyperbilirubinemia, respiratory distress syndrome, polycythemia and subsequent obesity and type 2 diabetes. Despite several international workshops and a lot of research there is still no unique approach to diagnose and treat diabetes in pregnancy. Who, when and how to screen and diagnose diabetes in pregnancy has been debated in the literature for so many decades and this debate seems to be endless. We present the evolution that screening and diagnosing diabetes in pregnancy has had over time. Besides many evidence of the benefits these procedures bring, health care providers still often prefer to use alternate criteria for this purpose. The myriad of maternal and fetal complications that could be avoided with an appropriate and simple screening procedure are ignored. Robust clinical trials such as the Hyperglycemia and Adverse Pregnancy Outcomes (HAPO) study have shown how harmful can even slightly altered blood glucose levels be, but it has been found a resistance in the adoption of the new criteria proposed after this and other trials by many diabetes organizations. These organizations state that these new criteria would increase the incidence of diabetes in pregnancy, would imply in longer term follow-up of these patients and would pose an economic problem; they also state that alerting too many people in order to benefit a relatively few potential diabetics would arise psychologic ill-effects. We think that health care providers should look for an uniformity in the screening and diagnosing diabetes in pregnancy based on evidence based medicine and not on specialists consensus.

## Introduction

Diabetes mellitus is a very ancient disease first described in the Egyptian Ebers papyrus around 1500 BC; written records of human pregnancy are still older. Although, the first description of diabetes in pregnancy was done by Bennewitz in 1824 in Germany [1]. He described a clinical case of a woman with intensive thirst and recurrent glycosuria in three successive pregnancies. One of her babies weighted almost 5,5 kg. Her urine contained a big amount of saccharine matter (about 60 g per 0,20 L). In 1846 a similar case was reported by Lever [2].

Before the discovery of insulin in 1922, infertility was well recognized in women with diabetes. The suggested causes of infertility present in these women were amenorrhea, uterus and Graafian follicles atrophy and malnutrition [3,4]. Few reports of conceptions in women with diabetes existed then; seven pregnancies in 114 women with diabetes [3], 55 in 427 women with diabetes of childbearing age [5], and four in 190 married women with diabetes [6]. After the discovery of insulin and its use initiation in 1923, the pregnancy rate increased by seven-fold in women with a short duration of the disease; women with a long duration of diabetes still remained sterile or with low conception rates for a long time.

In 1882, Duncan in London, reported the outcomes of pregnancy in 16 women with 22 pregnancies. High rates of maternal and perinatal mortality were present: more than 60% for the mothers and 47% for the newborns. The observations and the findings he had following these pregnancies allowed him to several conclusions such as: that diabetes may develop during pregnancy; diabetes may occur only during pregnancy, being absent in other times; diabetes may cease with the termination of pregnancy, recurring some time after birth; diabetes may develop soon after parturition; diabetes may not return in a pregnancy occurring after its cure; pregnancy may occur in the presence of diabetes; pregnancy and delivery may be apparently unaffected in its healthy progress by diabetes and finally that pregnancy is likely to be interrupted frequently by the fetus death [7].

Williams, Professor of Obstetrics in Baltimore, in 1909, reported 66 cases from the literature. Fifty-five patients had diabetes previous to the conception; nine patients developed diabetes after conception and in two the time of onset was not certain. The mortality rates were still high, being 27% at the time of delivery with around an additional 23% dying within two years after delivery. The perinatal mortality rates varied from 27-53% [8]. The principal focus of his manuscript was on the interpretation and the diagnostic role of glycosuria in pregnancy, because at that time the diagnosis of diabetes was based on the presence of sugar in the urine. He showed that if a woman’s urine had between 1 and 3 g /L of sugar, it was most likely to be a physiologic condition, but a higher concentration was suggestive of diabetes, particularly if present in early pregnancy or in the presence of symptoms. His study might have been the first prospective screening program for diabetes in pregnancy [8].

The presence of glycosuria during pregnancy and its role as diagnostic of asymptomatic diabetes was a strongly debated subject by that time. In 1856, the presence of physiological glycosuria in pregnancy and lactation was first described [9], and in 1877 different types of sugar were identified in the urine, being lactose the most frequently type of sugar found in the urine of pregnant women [10]. The incidence of true glycosuria varied from 10% to 100%; some authors believed that it represented true diabetes and others that it was a benign condition. The believe that it might represent true diabetes was based on the fact that many women that presented glycosuria had typical symptoms of diabetes such as polydpsia, polyuria, polyhydramnios and even adverse fetal outcomes [8].

The cause of glycosuria was unknown. Some suggested that it was alimentary (caused by a greater absorption of carbohydrates) or toxemic (caused by liver abnormalities). Brocard, in 1898 demonstrated by the first time that pregnant women were less tolerant to sugar compared to non-pregnant women; he has found the presence of glycosuria 2 hours after the ingestion of 50 g of glucose in 50% of pregnant women compared to 11% found in non-pregnant women [11]. Glycosuria was also found to be recurrent in successive pregnancies [11].

In order to solve this problem of classifying a woman as having or not diabetes based on the glycosuria levels, J.W.Williams recommended a follow-up of all mothers that presented glycosuria for possible complications of diabetes. He concluded that it was important to distinguish if the patient had a transient or a persistent glycosuria, to distinguish whether the sugar was lactose or glucose. If glycosuria appears late in pregnancy, is less than 2%, and not accompanied by symptoms, it is probably transient, of slight clinical significance and indicates the patient should be carefully watched. However, if glycosuria appears early in pregnancy and in large amounts, it represents a more serious condition, because it will make it difficult to diagnosis diabetes until after delivery. In cases of diabetes it will persist; the course of diabetes in pregnancy is variable, pregnancy may occur in women with diabetes or diabetes may withdrawn manifest during pregnancy and finally he suggested that if the amount of glycosuria is large and cannot be controlled, the induction of abortion or premature labor should be indicated, even if the patient does not show severe symptoms [8].

Between 1920 and 1930 many reports have described the presence of pancreatic abnormalities in stillborn infants from mothers with diabetes, mainly hypertrophy of Langerhans’ islands; which was suggested to occur as a consequence of glucose transfer from the mother to the fetus, to a poor maternal glucose control and the possible cause of severe neonatal hypoglycemia, that could be fatal in a few days after birth [4,12].

After the discovery of insulin, and its use during pregnancy, many reports of its efficacy were done by many authors [6,13-16]. Lambie in Edinburgh, in 1926, pertinently concluded that when diabetes appears for the first time in pregnancy, it usually manifests in the fifth or sixth month and exceptionally before the fourth or after the eighth month of gestation. He also suggested the 50 g oral glucose challenge test (OGCT) for calculating the ketogenic-antiketogenic balance [16]. Skipper in 1933, published a vast review of the literature in the use of insulin in pregnancy and found a dramatic improvement in maternal mortality and a modest impact on fetal and neonatal outcomes and survival [6]. He then concluded that the use of insulin has led to lower maternal mortality, but no reduction in fetal mortality; women with diabetes usually present glucose intolerance during the latter months of pregnancy; hypoglycemia is common in the puerperium and may have serious consequences including coma; if a woman with diabetes receives an adequate treatment, pregnancy should not be harmful; ketonuria is common in badly treated cases; the most important cause of fetal death is poor metabolic control, overdevelopment of the fetus and presence of congenital malformations; every pregnant woman with glycosuria should be investigated as possibly having diabetes because it may appear during pregnancy; a rigid control of diabetes through the evaluation of glycosuria is of great importance; cesarean section may be indicated when the fetus is overdeveloped; breast feeding should always be tried and sterilization should be considered in women with unstable diabetes and according to the number of children the patients already had [6]. Many of his conclusions are applied with some modifications and adaptations until today.

Miller in 1945 reported the first observations on obstetrical complications in the prediabetic period [17]. In the 1950s many risk factors for the development of abnormalities in carbohydrate metabolism in pregnancy were defined and the term gestational diabetes mellitus (GDM) became accepted [18-21]. Soon after, screening programs were proposed for the early detection of diabetes in pregnancy.

In 1949, Dr. Priscilla White working at the Joslin Clinic in Boston, wrote a paper and proposed the “White's Classification” that became a hallmark in the classification of diabetes and pregnancy. This classification was revised many times in order to separate those patients with GDM from those with pre-existing diabetes. An alphabetic list was added to the original classification that took into account the age of diabetes onset, diabetes duration and the presence of diabetes-related complications [22].

### Screening for hyperglycemia in pregnancy

In the 1960s, the screening for GDM was done by taking patients’ history alone. The increased obstetrical risk associated with GDM, was first described by Hoet in 1954 [23]. Soon after that the National Institutes of Health developed a program in the epidemiology of chronic diseases, and a center for their study was established in Boston, Massachusetts, under Hugh Wilkerson [24]. At that time the role of glycosuria in pregnancy was controversial, although most investigators agreed of the possibility that it could be the first indicator of the presence of diabetes mellitus.

Based on Hoet’s study [23] and in the observation of a large group of women who were followed-up by Dr. John B. O’Sullivan, Wilkerson and Remein [19] in 1957 proposed offering a 3-hour oral glucose tolerance test (OGTT) for patients presenting risk factors for diabetes such as family history of diabetes, gestational glycosuria and overdeveloped infants at birth. For women without known risk factors, they proposed determining a 1-hour blood glucose value after the ingestion of a 50 g glucose load. A value of 130 mg or more was considered abnormal and a 3-hour OGTT should be performed afterwards [19].

Jackson in 1960, wrote a review article stating that a temporary abnormality in glucose tolerance during pregnancy indicated a potentially permanent diabetes state in the mother [25]. He also defined different stages in the development of diabetes: prediabetes (patients with a retrospective diagnosis of diabetes and with significant presence of risk factors for its development); chemical diabetes (asymptomatic patients with abnormal glucose tolerance) and finally overt diabetes (symptomatic patients) [25].

In order to detect any degree of carbohydrate metabolism disorder early in pregnancy, several modifications were proposed for the OGTT like the use of intravenous tolbutamide by Unger and Madison in 1958 [26] and of cortisone some hours before the oral glucose load by Conn and Fajans in 1961 [27]. The obtained curves presented much higher values than those performed without any drug and the methodology was abandoned.

There was a great confusion with the criteria for the definition of diabetes during pregnancy and even outside of pregnancy, based on glucose tolerance tests, hampered by different methodology to determine blood glucose levels (Somogyi-Nelson and Folin-Wu in the USA and Henederman in Europe), by the concentration of glucose in the solution to be ingested and whether the determination of glucose levels should be done in venous or capillary blood [4]. The Somogyi-Nelson, Folin-Wu and Henederman assays, are not specific for glucose; they measure all reducing substances present in the whole blood and give results that are 15–20 mg/dl higher than assays that measure only glucose [4].

The controversy on how to screen and diagnose GDM was great. Using the OGTT criteria for nonpregnant subjects, in pregnant women, the incidence of diabetes was about one-third of the entire pregnant population. In order to solve this problem, O’Sullivan performed 100-g OGTTs in 752 mainly second- and third-trimester pregnant women and found with the statistician Claire Mahan the first, second, and third standard deviation upper limits for these glucose values [28]. These were the first statistically based criteria for assessing glycemic normality in pregnancy. Compared to those found in normal individuals they had higher upper-limit values at the 2nd and 3rd hour, consistent with an impaired glucose tolerance in pregnant compared with nonpregnant individuals. The O’Sullivan and Mahan criteria, became the standard for diabetes detection in pregnancy for the next decades, although they were originally formulated to predict type 2 diabetes in the future and not to predict maternal and fetal problems in the index pregnancy [28]. The values proposed by O’Sullivan and Mahan were: fasting, 110 mg/dl; 1-hour, 170 mg/dl; 2-hours, 120 mg/dl and 3-hours, 110 mg/dl (for Somogyi-Nelson method and venous blood). Two or more abnormal values were enough to diagnose an abnormal test [28].

These values selected by O’Sullivan and Mahan represented the mean plus two standard deviations because they believed that the more lenient the test, for example mean plus one standard deviation, the greater would be the prevalence of diabetes, resulting in a long term follow-up of these patients what would pose an economic problem. They also believed that alerting too many people in order to benefit a relatively few potential diabetics would arise psychologic ill-effects [28].

Many studies such as those conducted by Pedersen and Priscilla White, showing the importance of maternal glucose levels in the outcomes of pregnancy in women with diabetes have changed the focus of the importance of diagnosing and treating these women as early as possible, not only aiming to predict the risk of type 2 diabetes in the future, but also to prevent adverse outcomes with the mother and the fetus in the current pregnancy [22,29].

In 1979, the National Diabetes Data Group (NDDG) converted the values of whole blood glucose thresholds to those approximately 14% higher plasma glucose values, as most of the laboratory instruments started to report plasma glucose values instead of whole blood glucose [30].

Gradually antenatal screening for hyperglycemia in pregnancy became established but also different screening and diagnostic procedures became proposed, even in the same country. The increasing incidence of diabetes in the background population, the altering demographic changes in human reproduction, the increasing prevalence of obesity among many other factors, resulted in important variation in the reported prevalence. For this reason, a series of International Colloquia on Carbohydrate Metabolism in Pregnancy were conducted between 1973 and 1988, four of them held in Aberdeen in Scotland. All of them failed to reach a worldwide consensus on the dose of glucose to use, how it should be given and when blood glucose should be measured [31].

### Diagnosing hyperglycemia in pregnancy

#### The international workshops on gestational diabetes mellitus

Because of a growing disagreement in the best way to screen and diagnose diabetes in pregnancy Norbet Freinkel organized the First International Workshop on GDM in October 1979 in Chicago; another four would still come and also take place in Chicago. GDM was then defined as “carbohydrate intolerance of variable severity recognized for the first time in pregnancy”. The criteria used for the diagnosis were those established by O’ Sullivan and Mahan in 1964 [28,32,33]. It was then recommended reinforcement in research to achieve more accurate diagnosis, precisely define outcomes criteria, correlate outcomes with maternal variables and finally find more effective therapy alternatives to control blood glucose levels. It was also proposed that if a patient was at risk for glucose intolerance, a fasting plasma glucose or a random glucose at least 2 hours postprandial should be done. All women who had not been identified as having glucose intolerance before 24 weeks gestation, should be screened for GDM between 24–28 weeks gestation. A special attention should be given to those patients with a fasting plasma glucose level > 105 mg/dl. In cases of GDM, a close surveillance of the mother and the fetus should be done; nutritional counseling, including advice to limit intake of concentrated sweets and insulin therapy should be established if diet alone failed to maintain a fasting plasma glucose < 105 mg/dl and a 2-hour postprandial < 120 mg/dl; oral hypoglycemic agents were not recommended. A strict control of blood glucose levels showed to be important in reducing fetal and perinatal morbidity and mortality [33].

The Second International Workshop on GDM was held in October 1984. The definition of GDM developed at the First Workshop was confirmed, adding that “the definition applies irrespective of whether or not insulin is used for the treatment or if the condition persists after pregnancy. It does not exclude the possibility that the glucose intolerance may have antedated the pregnancy” [34]. In terms of GDM detection, it was determined that all pregnant women should be screened for glucose intolerance, since selective screening based on clinical attributes or past obstetric history is inadequate. This screening should be performed by glucose measurement between 24–28 weeks gestation in women not identified as having glucose intolerance before the 24^th^ gestation week. A 50 g oral glucose challenge test (OGCT) for screening was proposed, regardless of last meal or time of the day, and a venous plasma glucose cutoff of ≥ 140 mg/dl on a sample obtained one hour after the glucose load was considered abnormal. For diagnostic purposes it was recommended to continue the utilization of 100 g OGTT and its interpretation according to diagnostic criteria of O’Sullivan and Mahan. Capillary blood measurement should not be used for diagnostic purposes. The measurement of glycated hemoglobin was also not considered a sensitive diagnostic indicator for GDM. In terms of management of GDM, those patients with fasting and potprandial hyperglycemia should be considered at greater risk for intrauterine death or neonatal mortality; they must undergo careful antepartum fetal surveillance. It was also mentioned by the first time that impaired carbohydrate tolerance may develop in macrosomic offspring. The nutritional counseling comprehended limitation of sucrose intake, monitoring of maternal weight, a caloric intake equivalent to that of nondiabetic women of normal weight but not so restrictive in calories. A program of moderate exercise was also recommended [34].

The blood glucose levels should be monitored, and if dietary management does not consistently maintain fasting plasma glucose < 105 mg/dl and/or a 2-hour postprandial plasma glucose < 120 mg/dl on two or more occasions within a two week interval, insulin should be initiated, accompanied by self-monitoring of blood glucose; breastfeeding should be encouraged. Finally, it was reinforced that more than half of women with GDM will develop permanent diabetes. In order to detect diabetes early, an evaluation with a 2-hour, 75 g OGTT should be performed at the first postpartum visit. Regular physical activity should be encouraged to these patients [34].

The Third International Workshop on GDM happened in November 1990. The previous definition of GDM was confirmed. Screening and diagnostic criteria were also confirmed but with some modifications: Plasma glucose levels ≥ 200 mg/dl outside of formal OGTT, or fasting glucose ≥ 140 mg/dl suggests a diabetic state, warranting further investigation. A proportion of patients who meet recommended criteria for GDM have screening levels < 140 mg/dl and consequently the detection of GDM requires a substantial increase in the number of full OGTT performed. Also for diagnostic purposes, it is to mention that adjustments for conversion of whole blood glucose concentrations to equivalent plasma glucose values may overcorrect glucose levels; for this reason it is inadvisable to introduce minor corrective modifications. One single abnormal OGTT value may merit further evaluation since it may be associated with increased morbidity. Fixed diagnostic criteria were suggested for all populations. Macrosomia could be clinically estimated by fetal size and asymmetric growth identified by ultrasonography, and an earlier intervention could improve this outcome. In terms of long-range implications, it was emphasized that babies born to mothers with GDM present an increased risk of overt diabetes later in life and an increased likelihood of obesity, glucose intolerance and neurobehavioral and developmental abnormalities at birth and during childhood [35].

In March 1997 happened the Fourth International Workshop on GDM. The previous definition of GDM was confirmed. It was proposed and recommended a screening strategy to identify women at low-risk (belonging to an ethnic group with a low prevalence of GDM, having no known diabetes in first-degree relatives, aged < 25 years, presenting normal weight before pregnancy and at birth, no history of abnormal glucose metabolism or of poor obstetric outcome) who would not need evaluation; average risk (should perform blood glucose testing at 24–28 weeks using either a two-step procedure with a 50 g OGCT followed by a diagnostic OGTT in those meeting the threshold value in the OGCT of ≥ 140 mg/dl, or a one-step procedure with an OGTT performed on all subjects) as shown in Table 1, and high risk (those with at least one or more of these risk factors: marked obesity, strong family history of type 2 diabetes, previous history of GDM, impaired glucose metabolism, glucosuria or belonging to high-risk ethnic groups such as Hispanic, African, Native American, South or East Asian and from Pacific Islands, or of Indigenous Australian ancestry) it was recommended universal screening or diagnostic testing using the Carpenter and Coustan criteria for interpretation of the 100 g OGTT, with new cutoff values: fasting 95 mg/dL, 1h 180 mg/dL, 2h 155 mg/dL, 3 h 140 mg/dL, and also a 75 g 2-hours OGTT with the above criteria. They should perform blood glucose testing as soon as feasible. If GDM is not diagnosed, blood glucose testing should be repeated at 24-28 weeks or at any time a patient has symptoms or signs suggestive of hyperglycemia [36]. For the first time it was recommended the use of ultrasound to detect congenital anomalies in patients with GDM diagnosed in the first trimester or who presented with fasting glucose concentrations > 120 mg/dL [36].

**Table 1:** Screening and diagnosis of GDM in a one or two-step approach according to ADA

**SCREENING**		
**Single step**	**OGTT 100 or 75g**	**For average and high risk pregnant 24**^**th**^**-28**^**th **^**gestation weeks**
**Two steps**	**OGCT 50g If 1-hour≥ 140 mg/dl Perform an OGTT 100g**	**For all pregnant women 24**^**th**^**-28**^**th **^**gestation weeks**
**DIAGNOSIS**	**OGTT 100g**	**OGTT 75g**
**FASTING**	**95 mg/dl**	**95 mg/dl**
**1-hour**	**180 mg/dl**	**180 mg/dl**
**2-hours**	**155 mg/dl**	**155 mg/dl**
**3-hours**	**140 mg/dl**	**-**

Criteria for GDM diagnosis= 2 altered values.

75 g OGTT does not include the 3-hour value.

A carbohydrate-rich diet with more than 150 g/ day/ 3 days before the test.

Patients should be seated and do not smoke during the test.

Some new therapeutic interventions were proposed during pregnancy with GDM such as: ideal glycemic targets to prevent fetal risk should be lowered to capillary glucose levels of fasting ≤ 95 mg/dL, 1 h ≤ 140 mg/dL, and/or 2 h ≤ 120 mg/dL; the weight gain should be of ~ 7 kg for obese patients (BMI > 29 kg/m2) and greater weight gain of up to 18 kg for underweight patients (BMI < 19.8 kg/m2); it was recommended the use of glucose meters that store results electronically including postprandial testing as well as fasting and/or premeal testing; measurement of pre-breakfast urine ketone for patients on hypocaloric or carbohydrate-restricted diets. Insulin therapy was recommended with minimally antigenic insulin preparations for patients who fail glycemic goals or show signs of excessive fetal growth. Physical activity should be performed three times per week for at least 15 minutes [36].

In order to monitor fetal wellbeing it was recommended maternal fetal movement counting during the last 8–10 weeks of pregnancy; in patients requiring insulin, non stress testing from 32 weeks onward and at or near term in those requiring only dietary management. More complex fetal monitoring such as the biophysical profile or doppler assessment of umbilical cord blood flow may be considered when excessive or poor fetal growth are noted or there are complicating medical problems, such as preeclampsia. Fetal abdominal circumference measurements by ultrasound at 29–33 weeks gestation are useful in identifying a large subset of patients with maternal fasting glucose levels < 105 mg/dL who are at low risk for fetal macrosomia at term when managed with dietary therapy alone [36].

In terms of long-range implications and management after pregnancy, it was noted that the progression to type 2 diabetes within 5 years after the diagnosis of GDM was related to gestational age, severity of GDM at diagnosis, level of glycemia at first postpartum assessment, impairment of β-cell function, obesity, and further pregnancy. It was then recommended an evaluation of glucose tolerance in the mother 6–12 weeks postpartum with a 75 g OGTT; if postpartum testing does not indicate diabetes, fasting plasma glucose should be evaluated annually and in preparation for any future pregnancy. Patients should be instructed in lifestyle behaviors to reduce weight and increase physical activity to reduce the risk of subsequent diabetes; preconception counseling should be given to address appropriate contraception and women contemplating a future pregnancy should be advised to take supplementary folic acid to avoid risks of congenital malformations. An increased risk of obesity and abnormal glucose tolerance by puberty in offspring of women with GDM was identified, and lifestyle measures aimed at reducing or preventing obesity may decrease these risks. Breastfeeding should also be encouraged to reduce the risk of obesity and possibly diabetes in the offspring [36].

The Fifth International Workshop on GDM was held in November 2005, under the sponsorship of the American Diabetes Association (ADA). The meeting provided a forum for review of new information concerning GDM in the areas of pathophysiology, epidemiology, perinatal outcomes, long-range implications for the mother and her offspring, and management strategies as did the previous four International Worshops on GDM [37]. The issues regarding strategies and criteria for the detection and diagnosis of GDM were not reviewed or discussed in detail, since it was anticipated that the Hyperglycemia and Adverse Pregnancy Outcome (HAPO) study [38] would provide data that would adopt criteria for the diagnosis of GDM that would be based on perinatal outcomes. Thus, a motion to continue use of the definition, classification criteria, and strategies for detection and diagnosis of GDM that were recommended at the Fourth International Workshop was endorsed [36]. Minor modifications were done mainly in relation to metabolic assessments recommended after GDM. These assessments should be done as follows: a fasting or random plasma glucose 1–3 days after delivery, to detect persistent, overt diabetes; around the time of postpartum visit, a 75-g 2-hour OGTT for the postpartum classification of glucose metabolism; the OGTT should be repeated one year postpartum, then tri-annually and before another pregnancy in order to assess glucose metabolism. It was also recommended to measure a fasting plasma glucose annually [37].

After so many international workshops and several decades of research, there is still no unified global approach for GDM diagnosis [38-43], as seen in Table 2.

**Table 2:** Existing criteria for GDM diagnosis

	**Diagnostic test**	**Blood glucose values (mg/dl)**				**Diagnostic criteria**
		**fasting**	**1-hour**	**2-hours**	**3-hours**	
**National Diabetes Data Group, 1979**[30]	**100g OGTT-whole blood**	**105**	**190**	**165**	**145**	**2 or more values above limit**
**Carpenter e Coustan,1982**[38]	**100g OGTT- plasma glucose**	**95**	**180**	**155**	**140**	**2 or more values above limit**
**World Health Organization, 1998**[39]	**75g OGTT- plasma glucose**	**126**	**-**	**140**	**-**	**1 value above limit**
**Brazilian Health Ministry, 2002**[40]	**75g OGTT- plasma glucose**	**110**	**-**	**140**	**-**	**1 value above limit**
**ADA, 2004**[41]	**100g OGTT**	**95**	**180**	**155**	**140**	**2 or more values above limit**
**American Diabetes Association, 2009**[42]	**100g OGTT/ 75gOGTT**	**95**	**180**	**155**	**-**	**2 or more values above limit**
**Brazilian Health Ministry, 2002**[43]	**75g OGTT- plasma glucose**	**95**	**180**	**155**	**-**	**2 or more values above limit**
**ADA, 2011 (46) and IADPSG,2010**[45]	**75g OGTT- plasma glucose**	**92**	**180**	**153**	**-**	

#### The hyperglycemia and adverse pregnancy outcomes study

The objective of the Hyperglycemia and Adverse Pregnancy Outcome (HAPO) Study was to clarify the risk of adverse outcomes associated with different degrees of maternal glucose intolerance less severe than overt diabetes during pregnancy. Glucose tolerance was measured in approximately 25,000 women from nine different countries and fifteen different centers, in a heterogeneous, multicultural, ethnically diverse cohort of women at 24–32 gestation weeks. Positive associations were found between higher fasting, 1- and 2-h OGTT plasma glucose concentrations and birth weight >90th percentile and cord serum C-peptide >90th percentile, primary cesarean delivery, clinical neonatal hypoglycemia, preterm delivery, shoulder dystocia or birth injury, intensive neonatal care, hyperbilirubinemia, and preeclampsia, as well as with newborn adiposity [44].

The associations of maternal glycemia with perinatal outcomes were continuous with no obvious thresholds at which risks increased, it was evident that a consensus was required to translate these results into clinical practice. Many other issues had then to be addressed such as the importance to have all three OGTT glucose measurements (fasting, 1-, and 2-h-post load values) in the OGTT since the individual OGTT glucose measures were not highly correlated, and no single measure was clearly superior to each other in predicting the primary outcomes. It was necessary to find out the threshold at or above which the risk of adverse outcomes was too high.

#### The international association of diabetes and pregnancy study groups

The International Association of Diabetes and Pregnancy Study Groups (IADPSG) was formed in 1998 to facilitate collaboration between the various regional and national groups that have a primary or significant focus on diabetes and pregnancy. The IADPSG sponsored an “International Workshop Conference on Gestational Diabetes Diagnosis and Classification” in Pasadena, CA on June 2008 to initiate the process of a consensus development based on the data found in the HAPO study, associating maternal glycemia with perinatal and long-term outcomes in the offspring. Under the coordination from the Consensus Panel Steering Committee/Writing Group, the Panel reviewed further HAPO Study results provided by the HAPO Study Data Coordinating Center and the Consensus Panel has formulated the “Recommendations on the Diagnosis and Classification of Hyperglycemia in Pregnancy” which was soon after published, with new thresholds for the diagnosis of GDM [45]. It was then expected that this report would be considered by all of the major diabetes organizations and would serve as the basis for internationally uniform criteria for the diagnosis and classification of diabetes in pregnancy [45].

The new diagnostic criteria were soon adopted by many pre-eminent diabetes organizations such as the American Diabetes Association [46] and the Brazilian diabetes Society [47]. Despite the clear evidences that the HAPO study has shown on how harmful can even slightly altered blood glucose levels be, it has been found a resistance in the adoption of the new criteria by many diabetes organizations stating that these new criteria would increase the incidence of GDM from around 7% to 18.7%, and that the greater the prevalence of diabetes diagnosis, a longer term follow-up of these patients would be needed and would pose an economic problem, and also that alerting too many people in order to benefit a relatively few potential diabetics would arise psychologic ill-effects. These are the same arguments used by O’Sullivan and Mahan to select the upper standard deviation when they first described the OGTT in 1964. It seems that we did not have too much progress in the last decades.

## Conclusions

After several international workshops and many decades of research, there is still no unified global approach to GDM, as seen in Table 2. Most countries have their own diabetes associations each one with 1 to 3 diabetes societies as an International Diabetes Federation member [48]. These societies often have their own guidelines for GDM, which may be very similar or markedly different, and often, no guideline is proposed. The problem of GDM is the lack of an international consensus among these diabetes organizations. There is a wide diversity in the methods used in most countries due to multiple reasons. Health providers often prefer to use alternate criteria, follow the recommendation of a diabetes or health organization from another country and often there is disagreement between the country’s national diabetes organization, its local health society, and its regional obstetric organization, with each one recommending different approaches for screening and diagnosing GDM. It would be of interest of pregnant patients the formulation of unified universal guidelines for GDM. A consensus could be achieved with the evidence based gained from the data obtained in recent trials. It is time to an agreement about one global guideline for GDM.

## Abbreviations

HAPO study: The Hyperglycemia and Adverse Pregnancy Outcomes Study; OGCT: Oral glucose challenge test; GDM: Gestational diabetes mellitus; OGTT: Oral glucose tolerance test; NDDG: National Diabetes Data Group; IADPSG: The International Association of Diabetes and Pregnancy Study; ADA: American Diabetes Association.

## Competing interests

The authors declare that they have no competing interests.

## Authors’ contributions

Carlos Antonio Negrato and Marilia Brito Gomes drafted, reviewed and edited the manuscript. Both authors read and approved the final manuscript.

## References

[B1] BennewitzHGDe Diabete Mellito, gravidatatis symptomate1824MD Thesis, University of Berlin

[B2] LeverJCWGuy’s Hospital Report1847London3

[B3] LecorcheAnn de Gynecol et d’obst188524Paris257

[B4] MestmanJHHistorical notes on diabetes and pregnancyEndocrinologist20021222424210.1097/00019616-200205000-00010

[B5] Von NoordenCDie Die Zuckerkrankheit, Volume 41917Aufl

[B6] SkipperEDiabetes mellitus in pregnancy: A clinical and analytical studyQJM1933735380

[B7] DuncanJMOn puerperal diabetesTrans Obstet Soc Lond188224256

[B8] WilliamsJWThe clinical significance of glycosuria in pregnant womenAm J Med Sci190913712610.1097/00000441-190901000-00001

[B9] BlotCompt Rendus Soc Biol18835193

[B10] Hofmeister ZtschrFPhys Chemie18771101

[B11] BrocardLa glycosuria de al groaesser1898These de Paris

[B12] DubreuilGAnderodiasCompt Rendus Soc Biol19201331490

[B13] WalkerADiabetes mellitus in pregnancyProc Roy Soc Med1927–1928xxi1310.1177/003591572802100327PMC210201519986239

[B14] GrahamGA case of diabetes mellitus complicated by pregnancy treated with insulinProc Roy Soc Med1924xvii1021041998383210.1177/003591572401701028PMC2201739

[B15] RevenoWSInsulin in diabetic coma complicating pregnancyJAMA19238120012002

[B16] LambieCGDiabetes and pregnancyJ Obstet Gynecol Br Emp19263356360610.1111/j.1471-0528.1926.tb12131.x

[B17] MillerHCThe effect of the prediabetic state on the survival of the fetus and the birth weight of the newborn infantN Engl J Med194523337637810.1056/NEJM194509272331302

[B18] MossJMMullholandHBDiabetes and pregnancy with special reference to the prediabetic stateAnn Intern Med1951346786911481129110.7326/0003-4819-34-3-678

[B19] WilkersonHLCRemeinQRStudies of abnormal carbohydrate metabolism in pregnancyDiabetes195763243291344776110.2337/diab.6.4.324

[B20] CarringtonERShumanCRRearsonHSEvaluation of the prediabetic state during pregnancyObstet Gynecol1957966466910.1097/00006250-195706000-0000813431126

[B21] JacksonWPUCambridgeMADiabetes, prediabetes, mothers and babiesS Afr Med J19532779579713101907

[B22] WhitePPregnancy complicating diabetesAm J Med194956096161539606310.1016/0002-9343(49)90382-4

[B23] HoetJPCarbohydrate metabolism in pregnancy (translated from the French by F.D.W. Lukens)Diabetes195431121314187710.2337/diab.3.1.1

[B24] KnoppRHJohnBO’Sullivan: A Pioneer in the study of gestational diabetesDiabetes Care20022594394410.2337/diacare.25.5.94311978704

[B25] JacksonWPUPresent status of prediabetesDiabetes196093733781371851710.2337/diab.9.5.373

[B26] UngerRHMadisonLLA new diagnostic procedure for mild diabetes mellitus: evaluations of an intravenous tolbutamide response testDiabetes195874551359773910.2337/diab.7.6.455

[B27] ConnJWFajansSSThe prediabetic stateAm J Med19613183985010.1016/0002-9343(61)90023-713880869

[B28] O’SullivanJMahanCCriteria for the oral glucose tolerance test in pregnancyDiabetes19641327828514166677

[B29] PedersenJBrandstrupEFetal mortality in pregnant diabeticsLancet1956276076101332081910.1016/s0140-6736(56)90649-3

[B30] National Diabetes Data GroupClassification and diagnosis of diabetes mellitus and other categories of glucose intoleranceDiabetes1979281039105751080310.2337/diab.28.12.1039

[B31] HaddenDRSutherland HW, Stowers JMGlucose tolerance tests in pregnancyCarbohydrate Metabolism in Pregnancy and the Newborn1975Edinburgh: Churchill Livingstone1941

[B32] JovanovicLGestational Diabetes MellitusJAMA2001286202516251810.1001/jama.286.20.251611722247

[B33] FreinkelNJosinovichJFirst Workshop Conference on Gestational DiabetesDiabetes Care198033995016104569

[B34] Proceedings of the Second International Workshop-Conference on Gestational Diabetes MellitusDiabetes198534S211303996762

[B35] Third International Workshop Conference on Gestational Diabetes MellitusSummary and recommendationsDiabetes199140S2197201174825910.2337/diab.40.2.s197

[B36] MetzgerBECoustanDRSummary and recommendations of the Fourth International Workshop Conference on Gestational Diabetes MellitusDiabetes Care199821suppl 2B161B1679704245

[B37] MetzgerBEBuchananTACoustanDRDe LeivaADungerDBHaddenDRHodMKitzmillerJLKjosSLOatsJNPettittDJSacksDAZoupasCSummary and Recommendations of the Fifth International Workshop-Conference on Gestational Diabetes MellitusDiabetes Care200730S2S251S2601759648110.2337/dc07-s225

[B38] CarpenterMWCoustanDRCriteria for screening tests for gestational diabetesAm J Obstet Gynecol19821447768773714889810.1016/0002-9378(82)90349-0

[B39] AlbertiKGMMZimmetPZWHO ConsultationDefinition, diagnosis and classification of diabetes mellitus and its complications, Part 1: Diagnosis and classification of diabetes mellitus. Provisional report of a WHO consultationDiabet Med19981553955310.1002/(SICI)1096-9136(199807)15:7<539::AID-DIA668>3.0.CO;2-S9686693

[B40] ReicheltAJOppermannMLRSchmidtMIRecomendações da 2ª reunião do grupo de trabalho em diabetes e gravidezArq Bras Endocrinol Metab200246557458110.1590/S0004-27302002000500012

[B41] Professional Practice Committee/American Diabetes AssociationClinical practice recommendationsDiabetes Care200427Suppl. 1S51014693921

[B42] American Diabetes AssociationDiagnosis and classification of diabetes mellitusDiabetes Care2009321627

[B43] Brasil. Ministério da Saúde. Secretaria de Atenção à Saúde. Departamento de Ações Programáticas Estratégicas. Gestação de alto risco: manual técnico/Ministério da Saúde, Secretaria de Atenção à SaúdeDepartamento de Ações Programáticas Estratégicas20105ªBrasília: Editora do Ministério da Saúde302

[B44] MetzgerBELoweLPDyerARTrimbleERChaovarindrUCoustanDRHaddenDRMcCanceDRHodMMcIntyreHDOatsJJPerssonBRogersMSSacksDAHAPO Study Cooperative Research GroupHyperglycemia and adverse pregnancy outcomes. The HAPO Study cooperative research groupN Engl J Med2008358199120021846337510.1056/NEJMoa0707943

[B45] International Association of Diabetes and Pregnancy Study Groups Consensus PanelInternational Association of Diabetes and Pregnancy Study Groups Recommendations on the Diagnosis and Classification of Hyperglycemia in PregnancyDiabetes Care2010336766822019029610.2337/dc09-1848PMC2827530

[B46] American Diabetes AssociationDiagnosis and Classification of Diabetes MellitusDiabetes Care201134S62S692119362810.2337/dc11-S062PMC3006051

[B47] NegratoCAMontenegroRMJrMattarRZajdenvergLFranciscoRPPereiraBGSancovskiMTorloniMRDibSAViggianoCEGolbertAMoisésECFavaroMICalderonIMFusaroSPiliakasVDDiasJPGomesMBJovanovicLDysglycemias in pregnancy: from diagnosis to treatment. Brazilian consensus statementDiabetol Metab Syndr201022710.1186/1758-5996-2-2720416099PMC2867808

[B48] International Diabetes Federationhttp://www.idf.org. Accessed 02.23.13

